The article "Coupling coordination evaluation and driving path of digital economy and carbon emission efficiency in China: A fuzzy-set qualitative comparative analysis based on 30 provinces" was retracted in 2025. Reasons: concerns about the results or conclusions; concerns about the peer review; concerns about the authorship.

# Coupling coordination evaluation and driving path of digital economy and carbon emission efficiency in China: A fuzzy-set qualitative comparative analysis based on 30 provinces

**DOI:** 10.1371/journal.pone.0287819

**Published:** 2023-10-26

**Authors:** Zhou Li, Chen Xinlan, Mi Yixuan, Yang Guangming

**Affiliations:** 1 School of Business Administration, Chongqing Technology and Business University, Chongqing, China; 2 School of Management, Chongqing University of Technology, Chongqing, China; Shenzhen University, CHINA

## Abstract

Enhancing the level of coupling coordination between the digital economy (DIE) and carbon emission efficiency (CEE) is not only an inevitable choice for achieving the goals of energy conservation and emission reduction and promoting green development in China, but also a key path to implementing China’s “Double Carbon” strategy. Based on the relevant statistical data of 30 provincial-level regions in China from the period covering 2011 to 2019, this paper empirically analyzed the coupling coordination between the DIE and CEE and its influencing factors. In this study, an improved coupling coordination degree (CCD) model was used to evaluate the degree of the coupling and coordinated development of the DIE and CEE in provincial regions of China. Finally, based on the Technology-Organization-Environment (TOE) framework, a fuzzy-set qualitative comparative analysis (fsQCA) method was employed to identify the realization path of the coupling and coordinated development of the DIE and CEE from the perspective of configuration. The results demonstrated that the coupling coordination between the DIE and CCE in China demonstrated a gradual upward trend, and exhibited regional differences, showing a decreasing trend of east > middle > west. Regarding the influencing factors, no single influencing factor could act as a necessary condition for the high CCD, the coupling and coordinated development of the DIE and CEE is a multifactorial synergy. There were five paths for the high degree of coupling coordination between the DIE and CEE, which were divided into three types: organization-environment-led type, environment-led type, and technology-organization-led type. Furthermore, technological innovation level and industrial structure could substitute for one another in some conditions, and environmental regulation and economic development level were synchronized. These conclusions provide a theoretical basis for countries to formulate policies to promote the coupling and coordinated development of their DIE and CEE.

## 1. Introduction

Along with the rapid development and wide application of contemporary information technologies, such as the Internet, cloud computing, and big data, the digital economy came into being and is developing vigorously. In reality, China’s digital economy is developing rapidly. The data released in the Report on the Development of China’s Digital Economy (2022) shows that the scale of China’s digital economy reached 45.5 trillion yuan in 2021, with a nominal growth rate of 16.2%, and accounting for 39.8% of GDP [1, 2]. China has gradually entered the era of the digital economy. The rapid development of the digital economy is leading to profound changes in production, living, and governance methods, spawning new business forms and industries. Meanwhile, China is experiencing rapid development in urbanization and industrialization, leading to large consumption of energy and resources, high carbon emissions, and a series of problems including climate change that pose a great threat to nature and human beings [3, 4]. As shown from the statistical data in the BP Statistical Review of World Energy, China’s carbon emissions account for 29% of the world’s total carbon emissions [5], and China has been the world’s fastest-growing energy consumer for 19 consecutive years [6]. China ushered in a new era of low carbon led by the “Double Carbon” goal. To achieve its “Double Carbon” goal according to schedule, China’s 14th Five-Year Plan further proposes that the carbon emission intensity (carbon emission per unit GDP) be reduced by more than 65% by 2030 compared with 2005. As a new engine for regional development [7], the digital economy can improve the efficiency of resource allocation and reduce energy consumption and carbon emissions in traditional industries. It can be seen that the digital economy is an important booster for China to achieve the “Double Carbon” goal and a zero-carbon economy [8]. As a sustainable development model, low-carbon development, characterized by low energy consumption, low pollution, and low emissions, is the main economic and social development model of China in the future, and it will promote the low-carbon transformation of digital infrastructure, accelerate the process of industry digitization, and further enhance the scale of the digital industry [9]. In the context of the dual carbon strategy, the deep integration of the digital economy and low-carbon development has become an inevitable requirement and important support factor for achieving the goal of carbon emission reduction and promoting high-quality economic development. Carbon emission reduction is the key to achieving economic and environmental coordination and promoting sustainable development, and improving carbon emission efficiency is the key to achieving low carbon emissions. Therefore, the coupling coordination between the DIE and CEE is an urgent issue. What is the degree of coupling coordination between the DIE and CEE in China? Are there regional differences and spatial effects in the CCD of the DIE and CEE? Can China achieve the coupling and coordinated development of the DIE and CEE? These are the key scientific questions that this study needs to address. This paper took 30 provinces in China as the research objects, studied the degree of coupling coordination between the DIE and CEE through the construction of a measurement index system for the DIE and CEE, and further explored the factors affecting the coupling coordination between the DIE and CEE from a configurational perspective.

The article "Coupling coordination evaluation and driving path of digital economy and carbon emission efficiency in China: A fuzzy-set qualitative comparative analysis based on 30 provinces" was retracted in 2025. Reasons: concerns about the results or conclusions; concerns about the peer review; concerns about the authorship.

## 2. Literature review

Research on the DIE. The rapid development of the DIE has aroused widespread concern and discussion in academic circles. Extensive in-depth research on the DIE has been conducted by scholars in recent years, mainly focusing on three aspects: measurement methods, spatial layout, and driving forces. Firstly, in terms of the measurement methods. Scholars who have studied the measurement methods of the DIE include Ahmad et al. (2017), who applied direct measurement methods for research [10]; Zhang et al. (2022), using comprehensive evaluation method, who constructed a comprehensive evaluation index system from the three aspects of digital industry development foundation, digital innovation ability, and digital application level to measure the DIE at the urban level in China [11]; Li and Liu (2021), constructed an indicator system to measure the development level of the DIE by selecting evaluation indicators from the three dimensions of infrastructure construction, digital application, and digital industry development [12]; Luo et al. (2021) and Yang and Zhang (2019), designed the framework and compilation plan of China’s DIE satellite account [13, 14]. Others have evaluated the DIE in different regions and analyzed the impact of the DIE on the overall economy [15, 16]. Secondly, regarding the research on the spatial layout of the DIE, scholars have usually used the spatial Markov chain, the Dagum Gini coefficient, the Gini coefficient, a geographical detector, or exploratory spatial data analysis. In particular, they have paid attention to studying the spatial differentiation, spatial connection, and spatial spillover of the DIE and the influencing factors of its spatial pattern formation [12, 14]. In addition, Haita Wang et al. (2022) analyzed the spatial autocorrelation level and clustering type of China’s digital economy through Moran’s index method and the Getis-Ord General G tes [17]. Lastly, the existing empirical research on the driving force of the DIE shows that factors such as financial technology, economic growth, foreign investment, government support, labor resources, industrial structure, urban hierarchy, and information infrastructure have stimulated significant growth in the DIE in China [18, 19]. For example, a study by Wang et al. (2018) reveals that different dominant factors are driving the development of the digital economy in different regions [20].

The article "Coupling coordination evaluation and driving path of digital economy and carbon emission efficiency in China: A fuzzy-set qualitative comparative analysis based on 30 provinces" was retracted in 2025. Reasons: concerns about the results or conclusions; concerns about the peer review; concerns about the authorship.

Research on the CEE. Reducing carbon emissions is crucial to improving the ecological environment and creating a “green planet”. Hence, carbon emission reduction has increasingly received widespread attention from academia. There are many studies related to CEE, which can be classified into three categories: the measurement of CEE among different regions and industries, and the analysis of influencing factors of CEE. In general, most existing studies on the measurement of CEE focus on single-factor efficiency and multi-factor efficiency. For single-factor efficiency, the ratio of carbon dioxide (CO_2_) emissions to energy- or economy-related indicators is often selected as an evaluation indicator. For example, Li et al. (2021) analyzed that the change in intermediate input structure caused the change in the carbon intensity of the construction industry [21]. The multi-factor CEE fully considers the joint effects of labor, capital, energy, and other factors in the process of economic activities. The evaluation models commonly applied by relevant scholars mainly include improved models based on data envelopment analysis (DEA), including pure DEA [22], DEA window analysis [23], slack-based measure DEA (SBM-DEA) [24], super-efficiency SBM-DEA, and three-level edge DEA [25]. The DEA model was first proposed by the famous operations research scientists Charnes and Cooper in 1978 [26] and has now been widely used in the field of CEE [25, 27]. To further study the influencing factors of carbon emission efficiency, many scholars have combined the DEA model with the econometric model for analysis [28, 29]. Existing research shows that the impact of the economic scale, industrial structure, and openness on the CEE varies according to regional differences [30]. In addition, a study by Xiao et al. (2021) has found that the improvement of the economic development level can improve the CEE [31]. Li et al. (2019) conducted a separate study on the impact of urbanization on the CEE, and the results suggested that urbanization has had a positive impact on the CEE in the central and western regions of China, while the impact on the eastern region was not significant [32]. Cheng et al. (2017) empirically tested the impacts of different types of environmental regulations on carbon emissions using the dynamic space panel model and found that environmental regulations were conducive to carbon emission reduction [33]. In general, most scholars have focused on the impacts of economic development, openness, industrial structure, environmental regulation, and urbanization on the CEE.

The article "Coupling coordination evaluation and driving path of digital economy and carbon emission efficiency in China: A fuzzy-set qualitative comparative analysis based on 30 provinces" was retracted in 2025. Reasons: concerns about the results or conclusions; concerns about the peer review; concerns about the authorship.

Research on the impact of the DIE on CEE. The DIE is becoming an important engine to drive the development of low-carbon industries, promote the low-carbon transformation of the economy and society [34], and achieve the total amount of carbon emissions reduction [35], the intensity of carbon emissions reduction [36], the efficiency of carbon emission improvement [37]. Most scholars believe that the digital economy can achieve carbon emission reduction by promoting green technological progress [38], enhancing the efficiency of resource allocation [39], and promoting the upgrading of industrial structure [40]. Ning and Yang [41], empirically analyzed the impact of DIE on industrial CEE based on the provincial panel data of China, concluding that areas with the high level of DIE had higher CEE, and DIE played a significant role in promoting CEE. Cheng and Qu [42], using 282 Chinese urban panel data by improving various statistical methods of panel data, examined the extent and mechanism of the DIE’s impact on urban carbon emissions, and showed that DIE could significantly reduce carbon emissions through the rational layout of industrial structures. Furthermore, Ming et al. [43] applied the spatial panel Durbin model and the mediating effect model to empirically investigated the mechanism and influence of the DIE on carbon emission reduction and found that carbon emission reduction could be indirectly affected by the DIE through the transformation of energy structure, showing regional heterogeneity in the effect. There is still a lack of theoretical research and empirical analysis on the impact of the DIE on CEE, but existing relevant studies on the impact of the DIE, especially on carbon emissions, have laid the research foundation for this paper.

In summary, scholars have undertaken a large number of studies on the theoretical basis and mechanism of the DIE and CEE, but little attention is paid to the coupling coordination between the DIE and CEE, thus ignoring the potential links between the two systems. In addition to this, there is also a lack of systematic exploration of the dynamic evolution characteristics, spatial differences, and driving factors of the coupling coordination of DIE and CEE at the provincial level. The paper aims to reveal the realization of coordinated development of the DIE and CEE from the perspective of configuration. The structure of the paper is as follows: Section 2 is a literature review, which provides a comprehensive overview of scholars’ research on the DIE and CEE, and presents the innovation points of this paper. Section 3 is the research design, which introduces the research methodology, index system, influencing factors selection, and data source. Section 4 is an analysis of the CCD, including regional differences, spatial evolution characteristics, and spatial autocorrelation. Section 5 is a configuration analysis of the influencing factor of the CCD, which presents the driving path of the coupling and coordinated development of the DIE and CEE and the substitution relationship between conditions. Section 6 is the conclusions and suggestions, providing the findings of this research and proposing relevant policy suggestions. This paper aims to provide a scientific basis for enhancing the coupling coordination of China in terms of digitalization and low-carbon development.

The article "Coupling coordination evaluation and driving path of digital economy and carbon emission efficiency in China: A fuzzy-set qualitative comparative analysis based on 30 provinces" was retracted in 2025. Reasons: concerns about the results or conclusions; concerns about the peer review; concerns about the authorship.

## 3. Research design

### 3.1 Research methods

#### 3.1.1 Modified model of coupling coordination degree

The coupling coordination degree (CCD) can describe the dynamic relationship of development and coordination between systems [44]. The coupling coordination model, widely used in the fields of economics and geography, is suitable for describing the degree of interaction among different elements and systems, and it has obvious advantages for analyzing complex systems [45]. After summarizing the use and errors of the coupling coordination model, Wang Shujia et al. (2021) proposed a modified coupling coordination model that is more instructive than the traditional model [30]. Therefore, in this paper, we measured the CCD between the DIE and CEE by adopting the corrected coupling coordination model. The specific calculation formulas are as follows:

$$C=\sqrt{\left[1-\sum_{i>j,i=1}^{n}\sqrt{{\left(U_{i}-U_{j}\right)}^{2}}/\sum_{m=1}^{n-1}m\right]}\times {\left(\prod_{i=1}^{n}U_{i}/max\;U_{i}\right)}^{1/n-1}$$ (1)

$$T=\sum_{i=1}^{n}\alpha_{i}\times U_{i},\;\sum_{i=1}^{n}\alpha_{i}=1$$ (2)

$$D=\sqrt{C\times T}$$ (3)

Here, *C* is the CCD, where *C*∈[0,1]. Additionally, *U*_*i*_ and *U*_*j*_ represent the DIE development index and CEE index, respectively; *T* is the comprehensive evaluation index of the DIE and CEE; and *α*_*i*_ refers to the weight. Furthermore, *D* is the CCD of the DIE and CEE, where *D*∈[0,1]. A larger *D* value suggests that the coupling coordination between the two subsystems is better.

When *n* = 2, it is assumed that max *U*_*i*_ is *U*_2_:

$$C=\sqrt{[1-(U_{2}-U_{1})]\times U_{1}/U_{2}}$$ (4)

$$T=\alpha_{1}U_{1}+\alpha_{2}U_{2}$$ (5)

$$D=\sqrt{C\times T}$$ (6)

*α*_1_ and *α*_2_ indicate the contribution of DIE subsystem and CEE subsystem to the comprehensive system, respectively. We believe that the DIE and CEE systems is equally important, so this study takes *α*_1_ = *α*_2_ = 0.5. According to the calculated CCD and drawing on the existin relevant study [46, 47], this study constructed the evaluation standard of the coupling and coordination between the DIE and CEE to measure the level of coupling and coordinated development of the DIE and CEE better (**Table 1**).

The article "Coupling coordination evaluation and driving path of digital economy and carbon emission efficiency in China: A fuzzy-set qualitative comparative analysis based on 30 provinces" was retracted in 2025. Reasons: concerns about the results or conclusions; concerns about the peer review; concerns about the authorship.

**Table 1:** Evaluation standard for CCD classification.

CCD	Coupling effect level
0.00–0.20	Low coordination
0.20–0.40	Basic coordination
0.40–0.50	Moderate coordination
0.50–0.80	High coordination
0.80–1.00	Excellent coordination

#### 3.1.2 Spatial autocorrelation based on Moran’s index

Spatial autocorrelation analysis is an effective method that can characterize the degree of correlation among adjacent geographic units by considering both the location and attribute information of the research object synchronously. Moran’s index (Moran’s *I*) is the earliest method used to measure and describe the spatial distribution characteristics of variables and the degree of interdependence and mutual aggregation [48, 49]. In this paper, both global and local spatial autocorrelation models were employed to describe and visualize the spatial autocorrelation and spatial differentiation of the CCD development between the DIE and CEE at the province level in China. The global spatial autocorrelation model is used to reflect the overall spatial distribution of the CCD degree within the research scope and judge whether there is spatial agglomeration, which is expressed by global Moran’s *I* [50]. The specific formula is as follows:

$$I=n\times \sum_{i=1}^{n}\sum_{j\neq 1}^{n}W_{ij}(x_{i}-\bar{x})(x_{j}-\bar{x})/S^{2}\sum_{i=1}^{n}\sum_{j=1}^{n}W_{ij}$$ (7)

Here, *n* refers to the number of spatial units; *W*_*ij*_ represents the spatial weight matrix, built based on different criteria; *S*^2^ is the sample variance; *x*_*i*_ and *x*_*j*_ are the attribute values of *i* and *j*, respectively; and $\bar{x}$ is the mean value. In addition, the *Z* value from standard statistics is used to test the significance of Moran’s *I*. The value of the global Moran’s *I* is between –1 and 1. When *I* > 0, this indicates a positive spatial correlation in the CCD, that is, the high-value region of the CCD is adjacent to the high-value region, and the low-value region is adjacent to the low-value region; When *I* < 0, this indicates a negative spatial correlation in the CCD, that is, the high-value region of coupling coordination is adjacent to the low-value region. When *I* = 0, this indicates a random distribution, that is, there is no spatial correlation in the CCD.

The article "Coupling coordination evaluation and driving path of digital economy and carbon emission efficiency in China: A fuzzy-set qualitative comparative analysis based on 30 provinces" was retracted in 2025. Reasons: concerns about the results or conclusions; concerns about the peer review; concerns about the authorship.

The global spatial autocorrelation can only reflect the overall correlation state of the CCD of the study area, but cannot reflect the heterogeneity existing in a local area. Therefore, in this study, it is necessary to conduct a local spatial autocorrelation analysis. The local Moran’s *I* of the CCD was calculated and analyzed in combination with the LISA clustering map. The specific formula is as follows:

$$I_{i}=[\left(x_{i}-\bar{x}\right)/S^{2}]\times \sum_{j=1}^{n}W_{ij}(x_{j}-\bar{x})$$ (8)

Here, *I*_*i*_ is the local spatial autocorrelation coefficient; *I*_*i*_>0 suggests that there is spatial agglomeration; Conversely, *I*_*i*_<0 suggests that there is spatial dispersion. The local spatial association types between the target province and its neighbors can be divided into four quadrants of spatial clustering forms based on the values of local Moran’s *I* and characterized by their significance levels using the LISA significance test: high–high (H-H) clustering, high–low (H-L) clustering, low–low (L-L) clustering, low–high (L-H) clustering. Among them, H (L)-H (L) clustering indicates that the CCD of both the target province and its neighbors are at a high (low) level; H (L)-L (H) clustering indicates that the CCD of the target province is high (low), and the adjacent province’s CCD is low (high) [9, 51].

#### 3.1.3 Fuzzy-set qualitative comparative analysis

Qualitative comparative analysis (QCA) is a set-theoretic research method proposed by the American sociologist Charles C. Ragin in 1987 that can be used to analyze the causal complexity of social phenomena, combining the dual advantages of quantitative and qualitative analysis [52, 53]. Traditional econometric models treat elements as independent, making them unsuitable for studying complex causal interactions with many links [54]. Unlike conventional statistical analysis, QCA regards the case study as the conditional configuration and analyzes the causal relationship between different combinations of antecedent conditions from the perspective of configuration [55]. According to different data coding methods, QCA mainly includes three specific methods: clear-set qualitative comparative analysis (csQCA), fuzzy-set qualitative comparative analysis (fsQCA), and multi-value qualitative comparative analysis (mvQCA). Compared with csQCA and mvQCA, the fsQCA method utilizes affiliation calibration, thereby improving the study and more accurately explaining the complex causal relationships between conditional variable configurations and consequences [56]. Furthermore, this method applies to small and medium-sized samples [54, 57], especially when the country or region is taken as the analysis unit [58]. Which is more in line with the actual situation of this study. Therefore, the fsQCA method is very suitable for analyzing the driving path of the coordinated development of DIE and CEE.

The article "Coupling coordination evaluation and driving path of digital economy and carbon emission efficiency in China: A fuzzy-set qualitative comparative analysis based on 30 provinces" was retracted in 2025. Reasons: concerns about the results or conclusions; concerns about the peer review; concerns about the authorship.

The steps taken in the fsQCA to explore the factors influencing the coupling coordination between the DIE and CEE were as follows: calibration, necessity analysis, and sufficiency analysis [59]. This paper assumed that the coupling coordination between the DIE and CCE is comprehensively affected by various internal and external environmental factors. Therefore, fsQCA was employed to further explore the complex causal factors behind the coupling coordination between DIE and CEE from the perspective of configuration, finding multiple effective paths driving the coupling and coordinated development of the two subsystems.

### 3.2 Construction of index system

Referring to previous studies and following the selection principles of completeness, hierarchy, operability, and representativeness, we constructed a two-system comprehensive evaluation index system, as shown in **Table 2**. The digital economy is rich in connotation, not only it has a complex internal infrastructure, but also it is closely linked to social development [60]. Currently, there is no recognized evaluation system in academia for precise measurement of the DIE at the province level. Comprehensively integrating the existing research [11, 12, 61], this paper comprehensively considers digital infrastructure, digital industry development, digital finance development, and digital innovation capability based on the connotation and characteristics of DIE. Among them, as the technical carrier of digital economy development, digital infrastructure mainly reflects information network construction. In this paper, three indicators were selected for measurement: the cable line length, the number of mobile phone users, and the number of Internet broadband access users. Digital industry development mainly focused on the total amount of postal businesses, the total amount of telecom businesses, and urban unit employees in the information transmission and software and information technology services industry. For digital finance development indicators, we used the Digital Financial Inclusion Index of China, which is compiled by the *Digital Finance Research Center of Peking University*, including three indicators: coverage breadth of digital finance, usage depth of digital finance, and degree of digitalization [62]. Digital innovation leads to the transformation of industrial structure. In this article, technology market turnover accounted for the proportion of GDP, R&D funding input intensity, and the number of patents authorized was used for a comprehensive evaluation. To eliminate the impact of dimensional differences on each variable, we employed extreme value standardization to conduct dimensionless processing on the raw data. The specific formulas used are as follows:

$$X_{ij}^{\prime }=\left\{ \begin{array}{c} X_{ij}-{minX}_{.j}/{maxX}_{.j}-{minX}_{.j},X_{ij}\;\mathrm{is}\;\mathrm{positive}\;\mathrm{indicators}\\ {maxX}_{.j}-X_{ij}/{maxX}_{.j}-X_{ij},X_{ij}\;\mathrm{is}\;\mathrm{negative}\;\mathrm{indicators} \end{array}\right.$$ (9)

**Table 2:** Comprehensive evaluation indicator system for the DIE and CEE.

System layer	Criterion layer	Index layer	Indicator direction
**Digital economy level**	**Digital infrastructure**	Cable line length (km)	+
		Number of mobile phone users (10^4^ households)	+
		Number of Internet broadband access users (10^4^ households)	+
	**Digital industry development**	Total amount of postal business (10^8^ yuan)	+
		Total amount of telecom business (10^8^ yuan)	+
		Urban unit employees in information transmission and software and information technology services industry (10^4^ people)	+
	**Digital financial development**	Coverage breadth of digital finance	+
		Usage depth of digital finance	+
		Degree of digitalization	+
	**Digital innovation capability**	Technology market turnover accounted for the proportion of GDP (%)	+
		R&D funding input intensity (%)	+
		Number of patents authorized (pieces)	+
**Carbon emission efficiency**	**Input indicators**	Number of employees at the end of the year (10^4^ people)	+
		Capital stock (10^4^ people)	+
		Total amount of energy consumption (10^4^ tons)	+
	**Desirable output indicator**	GDP (10^8^ yuan)	+
	**Undesirable output indicator**	Total CO_2_ emissions (10^4^ tons)	−

Note: (+) positive dimensions; (−) negative dimensions.

The article "Coupling coordination evaluation and driving path of digital economy and carbon emission efficiency in China: A fuzzy-set qualitative comparative analysis based on 30 provinces" was retracted in 2025. Reasons: concerns about the results or conclusions; concerns about the peer review; concerns about the authorship.

Here, *i* represents the evaluation object; *j* represents the indicator; $X_{ij}^{\prime }$ and *X*_*ij*_ respectively denote the standardized and original value; and *maxX*_.*j*_ and *minX*_.*j*_ are the the maximum and minimum values of the indicator in the year of observation, respectively. The range of all indicator values after treatment is between 0 and 1 [63]. We standardized the original data and then calculated the information entropy value and utility value of each indicator using the entropy method. The specific calculation steps are as follow:

In the first step, calculate the share of indicator *j* in evaluation object *i*:

$$y_{ij}=X_{ij}^{\prime }/\sum_{i=1}^{n}X_{ij}^{\prime }$$ (10)

In the second step, calculate the information entropy *e*_*j*_:

$$e_{j}=-k\sum_{i=1}^{n}\left(y_{ij}\times \ln\;y_{ij}\right)$$ (11)

Generally, $k=\frac{1}{\ln n}>0,$ *e*_*j*_>0.

In the third step, calculate the information entropy redundancy *d*_*j*_:

$$d_{j}=1-e_{j}$$ (12)

In the fourth step, calculate the weight of each indicator *w*_*j*_:

$$w_{j}=d_{j}/\sum_{j=1}^{m}d_{j}$$ (13)

In terms of constructing the CEE index system, input and output variables were necessary for the evaluation of the CEE by the super-efficiency SBM model. Therefore, this paper selected evaluation indicators mainly in terms of the two aspects of input and output [64]. Drawing on existing research [65, 66], we selected capital stock, labor force, and energy consumption as the CEE input indicators. For the indicators, the capital stock was estimated using the perpetual inventory method, following the specific method used by Li and Zhang (2016) [67]. The labor force was estimated by the number of employees in each province at the end of the year, while the energy consumption was measured by the total amount of energy consumed by each province in a certain period (one year), taking standard coal as the statistical caliber. For the output indicators, the desirable output variable was measured by gross GDP, with GDP deflators used to convert the GDP of each year into constant prices to eliminate the impact of price factors. Here, 2011 was used as the base period. The undesirable output variable was measured by the total CO_2_ emissions. Since China has not released provincial and municipal CO_2_ emissions data, the CO_2_ emissions used in this paper were calculated based on the seven major fuels (coal, coke, gasoline, kerosene, diesel, fuel oil, and natural gas) and the National Greenhouse Gas Inventory Guidelines published by the 2006 Intergovernmental Panel on Climate Change (IPCC). The specific formula is as follows:

$${CO}_{2}=\sum_{i=1}^{7}{CO}_{2,\;i}=\sum_{i=1}^{7}E_{i}\times {CF}_{i}\times \frac{44}{12}$$ (14)

Here, *CO*_2_ is the estimated value of *CO*_*2*_ emissions, *E* represents the energy consumption, and *CF* denotes the carbon emission coefficient provided by the IPCC 2006 [68]. The molecular weights of *CO*_*2*_ and carbon are 44 and 22, respectively.

### 3.3 Influencing factors selection of CCD of the DIE and CEE

The coupling coordination between DIE and CEE is a complex process, and there are various factors that affect the coupling and coordinated development of the DIE and CEE. The coupling coordination refers to the elements and functions of the subsystems coordinating with each other, which jointly promote the evolution of the overall system to a higher level [69]. Based on the TOE framework proposed by Tornatizky and Fleischer, this study used the inductive method to identify six influencing factors of CCD in the three dimensions of technology, organization, and environment, and then constructed a configurational analytical framework to explore the driving factors of the coordinated development of the DIE and CEE (**Fig 1**).

The article "Coupling coordination evaluation and driving path of digital economy and carbon emission efficiency in China: A fuzzy-set qualitative comparative analysis based on 30 provinces" was retracted in 2025. Reasons: concerns about the results or conclusions; concerns about the peer review; concerns about the authorship.

**Fig 1:** Antecedent configuration analysis framework.

Technological conditions mainly stand for technological accessibility used to support the coordinated development of the DIE and CEE. In this study, the technological innovation level is regarded as technological factor affecting the coupling and coordinated development of the DIE and CEE. Technological innovation is a key manifestation of the DIE and an important driving force for the improvement of CEE. The higher the level of technological innovation in the organization, the more capable the organization of applying technology, and the greater the application of innovative technology [70]. In other words, provinces with high technological innovation levels are more likely to increase support for the development of DIE and improve the efficiency of carbon emission.

Organizational conditions include environmental regulation and industrial structure as two secondary conditions. Environmental regulation refers to the governmental policy-making and measures implemented by government to guide public behavior toward protecting the environment [71]. The government determines the development direction of the DIE and CEE by making relevant policies. In addition, the realization of low-carbon development goals largely depends on the local government’s decision-making preferences and the appropriate intensity of environmental regulation [72]. The adjustment and upgrading of industrial structure integrate resources and technology into the construction of low-carbon provinces, realize the optimal allocation of resources, and further improve the efficiency of resource utilization. Different industrial structures indicate that the development levels of provincial DIE and CEE are greatly different.

Environmental conditions mainly refer to the external environmental factors that affect the coupling and coordinated development of the DIE and CEE, which include three secondary conditions: economic development level, urbanization level, and degree of market openness. The economic development level is the basis for the development of the DIE. Provinces with high levels of economic development tend to pursue high-quality economic growth, and have the digital infrastructure for digital economic development [73]. Meanwhile, economic development provides financial and technical support for the low-carbon development of provinces, improves the CEE, and provinces with higher CEE are also more beneficial to development. The level of urbanization in a province is high, suggesting that its population quality and infrastructure are at excellent levels [74], which is beneficial to the coupling and coordinated development of the DIE and CEE.

The article "Coupling coordination evaluation and driving path of digital economy and carbon emission efficiency in China: A fuzzy-set qualitative comparative analysis based on 30 provinces" was retracted in 2025. Reasons: concerns about the results or conclusions; concerns about the peer review; concerns about the authorship.

### 3.4 Data sources

Considering the availability of data and the purpose of the research, this paper took 30 provinces in China during period of 2011–2019 as its research sample. Due to the unavailability of data on Tibet, Taiwan, Hong Kong, and Macao, these four regions were excluded. The digital inclusion fifinance index came from *Peking University Digital Inclusion Finance Index*, and the other data related to digital economy level were obtained from *the China Internet Network Information Center*, *the National Bureau of Statistics database (*http://data.stats.gov.cn/*)*, *the China Statistical Yearbook*, *and the statistical yearbooks of the individual provinces*. The input and output index data of the CEE were mainly collected from *the China Statistical Yearbook*, *the China Energy Statistical Yearbook*, *the China Environment Statistical Yearbook*, and *statistical yearbooks and statistical bulletins* of the various provinces. Some of the missing data were completed using the linear interpolation method.

## 4. Analysis of the coupling coordination between the DIE and CEE

### 4.1 Analysis on the CCD of DIE and CEE

Based on the comprehensive evaluation index system of the DIE and CEE, the degree of coupling coordination between the DIE and CEE in China’s provinces from 2011 to 2019 was calculated by Eqs (4–6), and the average CCD level of each province was classified as shown in **Table 3**. It was found that certain differences existed in the average CCD value of the DIE and CCE among China’s provinces. Three levels of moderate coordination, high coordination, and high-quality coordination existed, but most provinces fell into the two stages of moderate and high coordination. Among them, the number of provinces in the moderate coordination stage was 15, while 13 provinces were in the high coordination stage. Only Beijing and Guangdong were in the stage of high-quality coordination, while there were also no low- or basic-coordination provinces. On the whole, the CCD of DIE and CEE in all provinces of China was at or above the level of moderate coordination. Although there were no provinces with low or basic coordination, few provinces were in the stage of high-quality coordination. In the future, we should strengthen the construction of DIE and CEE in moderate- and high-coordination provinces and improve the level of coupling and coordinated development between the two subsystems to achieve coordinated regional development.

The article "Coupling coordination evaluation and driving path of digital economy and carbon emission efficiency in China: A fuzzy-set qualitative comparative analysis based on 30 provinces" was retracted in 2025. Reasons: concerns about the results or conclusions; concerns about the peer review; concerns about the authorship.

**Table 3:** Average CCD grades of China’s provinces from 2011 to 2019.

Grade	Low coordination	Basic coordination	Moderate coordination	High coordination	High-quality coordination
**Provinces**	No	No	Shanxi, Inner Mongolia, Jilin, Heilongjiang, Shanghai, Jiangsu, Zhejiang, Guangxi, Hainan, Guizhou, Yunnan, Gansu, Qinghai, Ningxia, Xinjiang	Tianjin, Hebei, Liaoning, Anhui, Fujian, Jiangxi, Shandong, Henan, Hubei, Hunan, Chongqing, Sichuan, Shaanxi	Beijing, Guangdong

To intuitively show the spatial distribution pattern of the level of coupling coordination between the DIE and CEE in 30 provinces, a visual representation of the type of coupling coordination between each province from 2011 to 2019 was carried out by applying ArcGIS 10.2 software. Considering the spatial differences in the coordinated development levels of the two and their more obvious evolutionary characteristics, this study selected the starting year and the intermediate year as the representative years for analysis, namely, 2011, 2014, 2016, and 2019 (**Fig 2**). In 2011, Beijing had the largest level of coupling coordination and had been in the high-quality coordination type at four-time nodes. Except for Jiangsu, Shanghai, Zhejiang, and Guangdong demonstrating the high coordination type, the remaining provinces were in the basic or moderate coordination type. The provinces in the western region were mainly in the basic coordination type, while those in the eastern region were mainly in the moderate coordination type. From 2011 to 2014, all provinces in the basic coordination type became the moderate coordination type, and there was no province in the basic coordination type. Tianjin and Shandong rose from moderate to high coordination type, and Guangdong became the high-quality coordination type. From 2014 to 2016, most provinces in China were in the moderate coordination type, and the number of provinces in the excellent coordination type increased from 2 in 2014 to 5. Sichuan, Hubei and Fujian became the high coordination type, while Jiangsu, Shanghai and Zhejiang increased to the high-quality coordination type. From 2016 to 2019, Tianjin decreased to the moderate coordination type. The number of provinces with high coordination type increased to 9, and the regional scope further extended to the central region. In summary, over time, the level of coupling coordination of all provinces increased to some extent, indicating that the relationship between the DIE and CEE is constantly improving. The CCDs of different provinces varied considerably and, on the whole, showed a spatial distribution pattern of eastern > central > western.

The article "Coupling coordination evaluation and driving path of digital economy and carbon emission efficiency in China: A fuzzy-set qualitative comparative analysis based on 30 provinces" was retracted in 2025. Reasons: concerns about the results or conclusions; concerns about the peer review; concerns about the authorship.

**Fig 2:** Spatial pattern of the CCD of DIE and CEE in China’s provinces.

### 4.2 Spatial autocorrelation analysis

To further explore the spatial agglomeration characteristics in the coupling coordination of the DIE and CEE in China as a whole, this paper calculated the global Moran’s *I* for the coupling coordination of the DIE and CEE from 2011 to 2019 based on Formula (7), and analyzed the overall spatial correlation characteristics of the coupling coordination (**Table 4**). It is observed that all the global Moran’s *I* values of coupling coordination were greater than 0, with a positive Z-score, and passed the significance test at a 1% level. The results suggested that there was a positive spatial correlation between the CCDs of 30 provinces during the study period. Numerically, the value of Moran’s *I* was distributed between 0.3199 and 0.3799, indicating a strong spatial correlation. Between 2011 and 2013, the value of Moran’s *I* decreased from 0.3504 to 0.3178, indicating that the positive spatial correlation of the CCD was gradually reduced in these years, probably due to the different economic bases, resource factors and ecological environment conditions of the provinces. Between 2014 and 2019, the value of Moran’s I continuously increased in fluctuation, and its significance rose year after year.

**Table 4:** Global Moran’s *I* of the CCD from 2011 to 2019.

Year	Moran’s I	Z value	P value
**2011**	0.3504	3.0606	0.002
**2012**	0.3494	3.0580	0.002
**2013**	0.3178	2.8057	0.005
**2014**	0.3270	2.8829	0.004
**2015**	0.3199	2.8362	0.005
**2016**	0.3779	3.2824	0.001
**2017**	0.3540	3.1200	0.002
**2018**	0.3747	3.2562	0.001
**2019**	0.3723	3.2357	0.001

To further detail the spatial correlation characteristics of the CCD of the 30 provinces from 2011 to 2019, we analyzed the local autocorrelation of coupling coordination with LISA clustering plots for 2011, 2014, 2016, and 2019 (**Fig 3**). As illustrated in Fig 3, from 2011 to 2019, there was only one type of agglomeration area in the coupling coordination between the DIE and CEE in China’s provinces: H-H clustering area. This type of area has a high level of coupling coordination with its surrounding areas, and the internal spatial difference is small. In 2011, 2016, and 2019, the H-H clustering area covered the same regions, including Jiangsu, Shanghai, and Zhejiang, forming an adjacent and mutually reinforcing linkage region. In 2014, under the radiation-driven effect of Jiangsu, Shandong entered the H-H clustering area and became a region with radiation capacity. In 2016, due to its limited radiation capacity and the reverse impact of other surrounding provinces, Shandong withdrew from the H-H clustering area. From the perspective of the overall evolution pattern, except for minor changes in 2014, there was no significant change in 2011, 2016, or 2019. In terms of spatial distribution, the H-H clustering areas were distributed in the east. During the study period, the spatial agglomeration effect of the coupling coordination between DIE and CEE in most provinces and cities in China was not significant, indicating that the synergy effect of the two subsystems needs to be strengthened. Accordingly, more H-H clustering areas should be built as soon as possible to give full play to the radiation and driving role of H-H clustering areas to improve the level of regional coupling coordination.

The article "Coupling coordination evaluation and driving path of digital economy and carbon emission efficiency in China: A fuzzy-set qualitative comparative analysis based on 30 provinces" was retracted in 2025. Reasons: concerns about the results or conclusions; concerns about the peer review; concerns about the authorship.

**Fig 3:** LISA clustering map of the CCD of the DIE and CEE in China.

## 5. Configuration analysis of the influencing factors of the CCD

### 5.1 Measurement and calibration of variables

#### 5.1.1 Variable selection and measurement

Result variable. Configuration analysis mainly studies the synergy and interdependence between conditional variables. According to the principle of fsQCA analysis, the variables are sorted into two categories: result and antecedent variables. The purpose of this study is to explore the driving path of the coordinated development of the DIE and CEE, thus the CCD of the DIE and CEE in the 30 provinces in China calculated by the coupling coordination model is the result variable in this paper.

Antecedent variables. According to Du Yunzhou et al. [55], for the study with medium-scale samples (10~50 cases), the number of ideal conditional variables should not exceed 8, and 4–7 should be preferred. In this paper, we take 30 provinces in mainland of China as research samples, belonging to the medium-scale sample, thus 6 conditional variables are selected to meet the sample requirements. This study finally considered economic development level, industrial structure, degree of opening up, technological innovation level, urbanization level, and environmental regulation as antecedent variables. The specific settings of each conditional variable were as follows: (1) Economic development level(ED). To eliminate the influence of the provincial population size on economic development, this study measured the level of economic development by calculating the natural logarithm of per capita GDP; (2) Industrial structure (IS). An advanced level of industrial structure is conducive to improving the efficiency of resource allocation and production. This paper used the proportion of added value of the secondary industry in the GDP to measure the industrial structure; (3) Degree of openness (OP),. this paper used the proportion of total import and export volume in the GDP of each province to directly measure the degree of market openness; (4) Technological innovation level (TI). Referring to the study of Xi Ji et al. (2018), we adopted the transaction volume of the technology market of each province as the index for directly measuring the technological innovation level [75]; (5) Urbanization level (UL). We selected the proportion of the urban population in the resident population to measure the level of urbanization. (6) Environmental regulation (ER), is a result of the government’s efforts to improve environmental governance and regulation. In this study, the proportion of completed investment in industrial pollution control among the GDP of each region was used to measure the environmental regulation intensity.

The article "Coupling coordination evaluation and driving path of digital economy and carbon emission efficiency in China: A fuzzy-set qualitative comparative analysis based on 30 provinces" was retracted in 2025. Reasons: concerns about the results or conclusions; concerns about the peer review; concerns about the authorship.

#### 5.1.2 Variable calibration

Calibration is a very crucial step in fsQCA analysis. Since fsQCA cannot analyze the panel data, and considering the contingency caused by using the data of a certain year, we used the average value of the 30 provincial regions from 2011 to 2019 by learning from the practice of Khedhaouria and Thurik. Since there was no obvious dividing point for the data, to ensure a relatively objective calibration, this paper referred to existing research [76] and defined 25%, 50%, and 75% of the quantiles of the raw data of six conditional variables and one consequence as full affiliation, crossover point, and full unaffiliation, respectively. At the same time, the direct calibration method was used to complete the fuzzy calibration of causal variables. The calibration anchor points and descriptive statistics of variables are shown in **Table 5**.

**Table 5:** Calibration results and descriptive statistical analysis of each variable.

Variable name		Anchor point			Descriptive statistical			
		Full affiliation	Crossover point	Full unaffiliation	Mean value	Standard deviation	Minimum value	Maximum value
**Result variable**	**CCD**	0.4608	0.5319	0.6077	0.5631	0.1410	0.1844	0.9950
**Condition variables**	**TI**	63.27	130.22	423.43	361.49	728.95	0.57	5695.28
	**ER**	0.0742	0.1	0.1658	0.1291	0.1269	0	1.1
	**IS**	0.3846	0.4324	0.4575	0.41	0.08	0.16	0.62
	**ED**	38603.66	43928.67	66138.06	54717	26271	16413	164220
	**UL**	50.89	55.95	62.68	58.19	12.23	35.03	89.6
	**OP**	1498.97	3769.96	8693.95	8850.99	14276.66	37.58	71763.36

### 5.2 Single-factor necessity analysis

A necessity test of a single variable is the premise of the conditional configuration analysis of fuzzy sets. When the consistency score of a single conditional variable is greater than 0.9, it is regarded as the necessary condition for the result variable [77]. In this paper, the fsQCA3.1 software was employed to test the necessary conditions of CCD. **Table 6** presents the results of the necessary conditions test. From Table 6, it can be seen that the consistency level of all condition variables was less than 0.9, indicating that all conditions antecedents cannot constitute the necessary conditions for achieving high or low CCD of the DIE and CEE. It was once again confirmed that the coupling and coordinated development of DIE and CEE was not determined by a single factor but was the result of multiple factors interacting and acting synergistically, with complex cause-effect relationships. Therefore, it is necessary to analyze the configuration effects of the six condition variables to further identify the differentiated conditional configurations leading to the high CCD.

The article "Coupling coordination evaluation and driving path of digital economy and carbon emission efficiency in China: A fuzzy-set qualitative comparative analysis based on 30 provinces" was retracted in 2025. Reasons: concerns about the results or conclusions; concerns about the peer review; concerns about the authorship.

**Table 6:** Results of the single-factor necessity test.

Condition variable	High CCD		Low CCD	
	Consistency	Coverage	Consistency	Coverage
**TI**	0.7888	0.8395	0.2713	0.2844
**~TI**	0.3276	0.3134	0.8469	0.7980
**ER**	0.3893	0.4082	0.6595	0.6813
**~ER**	0.6961	0.6748	0.4271	0.4079
**IS**	0.7333	0.7443	0.3888	0.3887
**~IS**	0.3977	0.3978	0.7442	0.7333
**ED**	0.7604	0.7854	0.3391	0.3451
**~ED**	0.3660	0.3599	0.7892	0.7644
**UL**	0.6651	0.6927	0.3801	0.3900
**~UL**	0.4143	0.4042	0.7005	0.6733
**OP**	0.8107	0.8573	0.2921	0.3043
**~OP**	0.3422	0.3292	0.8630	0.8179

*Note: “~” represents “non, no, or on the contrary.”

### 5.3 Sufficiency analysis of conditional configuration

A sufficiency analysis of condition configurations is the core of fsQCA, and it is used to explore the antecedent conditions or the combination of variables that lead to the results. Based on the research of Fiss [54], we set the consistency threshold of each configuration as 0.8 and the PRI (proportional reduction in inconsistency) threshold as 0.75. Meanwhile, there were only 30 cases included in the research, and the frequency value was set as 1 [54]. We adopted the fsQCA3.1 software to analyze results and obtained three types of solution: a complex solution, an intermediate solution, and a parsimonious solution. Following the general practice, this paper took the intermediate solution as the main reporting type and further distinguished the core condition and the marginal condition by combining it with the parsimonious solution. Condition variables that appeared in both the intermediate solution and parsimonious solution were considered core conditions. In contrast, condition variables that appeared only in the intermediate solution were considered marginal conditions. The configuration analysis results are presented in **Table 7**.

The article "Coupling coordination evaluation and driving path of digital economy and carbon emission efficiency in China: A fuzzy-set qualitative comparative analysis based on 30 provinces" was retracted in 2025. Reasons: concerns about the results or conclusions; concerns about the peer review; concerns about the authorship.

**Table 7:** Configuration of conditions for high CCD of the DIE and CEE.

Conditional variables	Organization-environment-led type		Environment-led type	Technology-organization-led type	
	H1a	H1b	H2	H3a	H3b
**TI**		X	O	O	O
**ER**		O		X	O
**IS**	O	O		O	O
**ED**	O	X	O	X	O
**UL**	O	X	O	X	X
**OP**	O	O	O	X	X
**Consistency**	0.9793	0.9565	0.9086	0.9854	0.9917
**Raw coverage**	0.4355	0.1019	0.5321	0.1343	0.0794
**Unique coverage**	0.0926	0.0437	0.1899	0.0774	0.0397
**Overall consistency**	0.9248				
**Overall coverage**	0.8213				

*Note: O represents the presence of a core condition, X represents the absence of a core condition, O represents the presence of an auxiliary condition, X represents the absence of an auxiliary condition, blank represents condition irrelevant to the outcome. This note also applies to the following tables.

It can be seen from **Table 7** that there were five configurations of conditions to achieve high CCD of DIE and CEE: configuration H1, configuration H2, configuration H3, configuration H4, and configuration H5. Consistency indicates the extent to which each configuration solution and each overall configuration solution are a subset of the results, and coverage represents the degree to which the configuration solution can explain the results [55]. The consistency values of these five configurations all exceeded the theoretical value of 0.8, indicating that they can be considered sufficient combinations of conditions to achieve the coupling and coordinated development of the DIE and CEE. The overall solution consistency was 0.9248, indicating that 92.48% of provinces had a high CCD in all cases that met the five condition configurations. The overall solution coverage was 0.8213, which means that these five configurations of conditions can explain 82.13% of the cases with high CCD. According to the different core characteristics of the antecedent conditions, the five configurations for achieving the coupling and coordinated development of the DIE and CEE can be divided into three types: organization-environment-led type (configuration H1a and H 1b), environment-led type (configuration H2), technology-organization-led type (configuration H3a and H3b).

Organization-environment-led type. Because in this configuration path, all antecedents came from both organizational and environmental aspects, and all condition variables were core conditions, we named it the “organization–environment-led type”, including configuration H1a and H1b. In configuration H1a, ED, IS, OP, and UL were the core conditions, and TI and ER were irrelevant for high CCD, which shows that the existence of ED, IS, OP, and UL can achieve the coupling and coordinated development of the DIE and CEE, and it will not be affected by TI and ER. This indicates that when a province with an optimized industrial structure, strong economic development and market openness, and a high level of urbanization, can achieve a high degree of coupling coordination between the DIE and CEE regardless of its TI and ER. This configuration explained 43.55% of the cases of high CCD; approximately 9.26% of the cases of high CCD could only be explained by this configuration. Typical provinces that corresponded to configuration H1a included Jiangsu, Zhejiang, Guangdong, Shandong, and Hubei, which are mainly located on the east coast of China. In configuration H1a, TI, ER, IS, and OP served as the core conditions, while ED and UL were the auxiliary conditions. Configuration H1b shows that the combination of the presence of ER, IS, and OP, in the absence of TI, ED, and UL, can generate sufficient conditions for the coupling and coordinated development of the DIE and CEE. This indicates that strong environmental regulation and market openness, and optimized industrial structure, along with low levels of technological innovation, economic development, and urbanization, can lead to a high CCD of the DIE and CEE. This configuration explained approximately 10.19% of cases with high CCD, and approximately 4.37% of cases with high CCD could only be explained by this configuration. Typical case that fits configuration H1b was Shanxi, which is in the northwest of China.

The article "Coupling coordination evaluation and driving path of digital economy and carbon emission efficiency in China: A fuzzy-set qualitative comparative analysis based on 30 provinces" was retracted in 2025. Reasons: concerns about the results or conclusions; concerns about the peer review; concerns about the authorship.

Environment-led type. Because in this configuration path, all the core conditions only came from the environmental aspect, we named it the “environment-led type”, with only one configuration H2. In configuration H2, ED, OP, and UL were the core conditions; TI was the marginal condition; ER and IS were irrelevant for high CCD. Configuration H2 shows that considering ED, OP, and UL as the core driving forces, supplemented by TI, can achieve a high CCD of the DIE and CEE. This indicates that high levels of technological innovation and urbanization, strong economic development, and market openness, can together lead to the coupling and coordinated development of the DIE and CEE. This path explained approximately 53.21% of the cases of high CCD, and approximately 18.99% of the cases of high CCD could only be explained by this path. We found that configuration H2 had the highest values of raw coverage, and unique coverage among the five configurations, indicating that configuration H2 was the primary configuration for provinces to achieve high CCD of the DIE and CEE. The cases in configuration H2 included provinces not only in the eastern coastal areas of Jiangsu, Guangdong, Tianjin, Zhejiang, and Shandong, but also in the central region of Hubei.

The article "Coupling coordination evaluation and driving path of digital economy and carbon emission efficiency in China: A fuzzy-set qualitative comparative analysis based on 30 provinces" was retracted in 2025. Reasons: concerns about the results or conclusions; concerns about the peer review; concerns about the authorship.

Technology-organization-led type. In this configuration path, the core conditions all came from two aspects of technology and organization, so we named it the “technology-organization-led type”, including two configurations: H3a and H3b. In configuration H3a, the core conditions were the existence of IS and TI; the marginal conditions were the absence of ED, OP, UL, and ER. Configuration H3a showed that provinces with an optimized industrial structure and a high level of technological innovation, along with low levels of economic development, market openness, and urbanization, could achieve a high CCD of the DIE and CEE, in which IS and TI played central roles, while the other conditions play auxiliary roles. This configuration explained approximately 13.43% of cases with high CCD, and approximately 7.74% of cases with high CCD could only be explained by this configuration. Typical cases that correspond to configuration H3a was Anhui, which is located in the east of China In configuration H3b, the core conditions were the existence of IS and TI; the marginal conditions were the existence of ED and ER, and the absence of OP and UL. H3b shows that the combination of the presence of TI, IS, ED, and ER, in absence of OP and UL, can lead to a high CCD of the DIE and CEE. This indicates that provinces with high levels of technological innovation and economic development, optimized industrial structure, and strong environmental regulation, along with low levels of market openness and urbanization, could lead to the coordinated development of the DIE and CEE. This configuration explained approximately 7.94% of the cases of high CCD, and approximately 3.97% of the cases of high CCD could only be explained by this configuration, with the lowest raw coverage and unique coverage among all of the configurations, which indicated that configuration H3b was the rarest path for provinces to achieve high CCD of the DIE and CEE. Typical case for this configuration was Henan, which is located in central China.

### 5.4 Horizontal analysis of antecedent conditions

After analyzing the conditions’ configurations, we can further identify the mutual substitution relationships between different conditions through a horizontal comparison of different configurations. The combined comparison of the five configurations showed that as a core element, the presence of IS appeared in four configurations (configurations H1a, H1b, H3a, and H3b) that achieved a high CCD of the DIE and CEE, indicating that IS significantly affects the coordinated development of the DIE and CEE.

The article "Coupling coordination evaluation and driving path of digital economy and carbon emission efficiency in China: A fuzzy-set qualitative comparative analysis based on 30 provinces" was retracted in 2025. Reasons: concerns about the results or conclusions; concerns about the peer review; concerns about the authorship.

By analyzing the similarities and differences of configurations H1a and H2, which achieve a high CCD of the DIE and CEE, it can be found that TI and IS can replace one another, and the substitution relationship is shown in **Fig 4**. Provinces with high levels of economic development, urbanization, and market openness, can achieve the coordinated development of the DIE and CEE by improving the level of technological innovation (H1a) or optimizing industrial structure (H2). Technological innovation can provide technical support for the coupling and coordinated development of the DIE and CEE; however, industrial structure can integrate resources and technology into the development of the DIE and the improvement of CEE, and further promote the coupling and coordinated development of the DIE and CEE. Therefore, TI and IS can be substituted for each other under certain conditions.

**Fig 4:** The potential substitution relationships between TI and IS.

In the given conditions, ER and ED were synchronous. It can be seen by comparing configurations H3a and H3b that it is the simultaneous presence or absence of ER and ED that can lead to high CCD of the DIE and CEE under the presence of TI and IS but with the absence of UL and OP.

## 6. Conclusions

Obtaining an accurate understanding of the coupling and coordination relationship between the DIE and CEE and its influencing factors is the premise of promoting the coupling and coordinated development of the economic society and ecological environment. Based on 30 provincial-level regions in China from 2011 to 2019, this study measured the CCD of the DIE and CEE by employing the modified CCD model and analyzed the spatial correlation between the two subsystems using Moran’s I. Furthermore, based on the TOE framework, fsQCA was applied to further explore the linkage effects and driving mechanisms of technical, organizational, and environmental factors on the CCD, revealing the realization path of the coupling and coordinated development of the DIE and CEE. The main conclusions were as follows: Firstly, the CCD of the DIE and CEE of all provinces exhibited an overall increasing trend to some extent, indicating that the relationship between the DIE and CEE was constantly improving, and there were great differences in the CCD of the DIE and CEE between the different provincial regions in China. Moreover, from a spatial perspective, the CCD of China’s DIE and CEE was high in the east and low in the west, showing a spatial distribution pattern of east > middle > west. Secondly, technological, organizational, and environmental conditions could not independently constitute the necessary condition for high CCD of the DIE and CEE, but the multiple concurrencies of them formed a diversified condition configuration that could attain a higher level of the coupling and coordinated development of the two subsystems, and the configuration paths of achieving a high CCD of the DIE and CEE had the characteristics of equivalence and multiple concurrencies. Thirdly, there were five paths that led to a high CCD of the DIE and CEE, which could be divided into three types: organization-environment-led type, environment-led type, and technology-organization-led type. Here, IS were the conditions in the four paths, which indicated that compared with other antecedent conditions, IS played a crucial role in the coupling and coordinated development of the DIE and CEE. Finally, under certain conditions, TI and IS could be replaced by each other to achieve the coupling and coordinated development of the DIE and CEE. Moreover, antecedent conditions of ER and ED were synchronous. The conclusions provide a new perspective to understand the path of achieving the coupling and coordinated development of the DIE and CEE, providing a theoretical basis for China and other developing countries to implement digital and low-carbon development strategies.

The article "Coupling coordination evaluation and driving path of digital economy and carbon emission efficiency in China: A fuzzy-set qualitative comparative analysis based on 30 provinces" was retracted in 2025. Reasons: concerns about the results or conclusions; concerns about the peer review; concerns about the authorship.

Based on the conclusions of this study, the following policy suggestions are put forward to promote the coupling and coordinated development of the DIE and CEE. Firstly, the opportunity for digital development should be grasped to accelerate the development of the DIE. China should closely follow the wave of digital development and continue to promote the development of the DIE by accelerating the breakthrough of digital technology, cultivating digital talent, and strengthening the construction of digital infrastructure. Secondly, cooperation between regions should be strengthened, and the overall level of coupling and coordinated development should be improved. China should adhere to the domestic cycle, promote healthy competition among regions, break the policy system and regional barriers, and formulate trans-regional cooperation and mutual assistance development strategies. The regions with a high degree of coordinated development in the east should provide reasonable assistance to the regions with a low degree of coordinated development in the center and west to promote the coordinated development of the eastern, central, and western regions. Thirdly, the realization paths of the coupling and coordinated development of the DIE and CEE have multiple concurrency. Regional governments should, based on their existing characteristics, focus on the adaptation of multiple conditions from an overall perspective, formulate policies according to their existing resource endowments and local conditions, and choose the appropriate driving path to promote the coupling and coordinated development of the DIE and CEE.

The article "Coupling coordination evaluation and driving path of digital economy and carbon emission efficiency in China: A fuzzy-set qualitative comparative analysis based on 30 provinces" was retracted in 2025. Reasons: concerns about the results or conclusions; concerns about the peer review; concerns about the authorship.

Compared with existing studies, the main contributions of this study have the following three aspects. Firstly, base on accurately understanding the connotation of DIE and CEE and drawing on existing research, this study established the evaluation index systems of the DIE and CEE for provincial regions in China, and then the modified CCD model and spatial autocorrelation model was used to evaluate and analyze the degree of coupling coordination and spatiotemporal characteristics between the DIE and CEE to comprehensively grasp the association and dynamic evolution trend of coupling coordination, which is a theoretical supplement to the existing research on DIE and CEE and expands the idea of studying DIE and CEE from the perspective of coupling. Secondly, this study selected six elements affecting the coupling coordination between the DIE and CEE from the TOE research framework and proposed an integrated analysis framework, which extends the scope of application of the TOE framework theory to a certain degree. Finally, this study adopted the fsQCA method to identify the driving path of the coupling and coordinated development of the DIE and CEE from a configurational perspective, and further analyzed the mutual substitution relationship between conditions through the comparison of different configurations, which breaks through the traditional statistical technique based on independent variables and one-way linear influence relationship.

There are some limitations in this study that need to be addressed in future research. First, we attempted to establish a comprehensive evaluation index system for the DIE and CEE, which may not be comprehensive enough due to the limitation of the public data acquisition. In the further, the construction of an indicator system can be improved and enriched by choosing appropriate indicators or comprehensive indicators to assess the CCD of the DIE and CEE more accurately. Second, although the TOE framework applied in this study covered the technological, organizational, and environmental factors influencing the degree of coupling coordination between the DIE and CEE, there were only six antecedent conditions selected due to the limitation of fsQCA on the number of condition variables. In the subsequent studies, more influencing factors of the coordinated development of the DIE and CEE should be incorporated into the model through factor analysis or principal component analysis. Third, in the study, we used static data to reveal the driving paths of the coordinated development of the DIE and CEE. In the future, the dynamic evolution of driving paths can be revealed with the combination of QCA and other analysis methods.

The article "Coupling coordination evaluation and driving path of digital economy and carbon emission efficiency in China: A fuzzy-set qualitative comparative analysis based on 30 provinces" was retracted in 2025. Reasons: concerns about the results or conclusions; concerns about the peer review; concerns about the authorship.

## Supporting information

S1 Table **A.** Total CO2 emissions of 30 provinces in China (2011–2019). **B.** CCD values of the DIE and CEE in China (2011–2019).
(ZIP)

S1 Dataset Raw data (2011–2019). (XLSX)
